The article "BMP2 secretion from hepatocellular carcinoma cell HepG2 enhances angiogenesis and tumor growth in endothelial cells via activation of the MAPK/p38 signaling pathway" was retracted in 2022. Reasons: duplicated images; unreliable results or conclusions.

# BMP2 secretion from hepatocellular carcinoma cell HepG2 enhances angiogenesis and tumor growth in endothelial cells via activation of the MAPK/p38 signaling pathway

**DOI:** 10.1186/s13287-019-1301-2

**Published:** 2019-08-06

**Authors:** Peng-Cheng Feng, Xing-Fei Ke, Hui-Lan Kuang, Li-Li Pan, Qiang Ye, Jian-Bing Wu

**Affiliations:** Department of Oncology, The Second Affiliated Hospital of Nanchang University, No. 1, Minde Road, Donghu District, Nanchang, 330006 Jiangxi Province People’s Republic of China

**Keywords:** BMP2, MAPK/p38 signaling pathway, Tumor growth, Angiogenesis, Hepatocellular carcinoma

## Abstract

**Background:**

Hepatocellular carcinoma (HCC) is one of the most common tumors globally, with varying prevalence based on endemic risk factors. Bone morphogenetic protein (BMP) exhibits a broad spectrum of biological activities in various tissues including angiogenesis. Here, this study aimed to investigate the mechanism of BMP2 in HCC by mediating the mitogen-activated protein kinase (MAPK)/p38 signaling pathway.

**Methods:**

BMP2 expression was quantified in HCC and adjacent tissues. BMP2 gain- and loss-of-function experiments were conducted by infection with lentivirus over-expressing BMP2 or expressing shRNA against BMP2. The angiogenesis was evaluated with HepG2 cells co-cultured with ECV304 cells. SB-239063 was applied to inhibit the activation of the MAPK/p38 signaling pathway so as to identify the significance of this pathway in HCC progression. Finally, in vivo experiments were conducted to identify the role of BMP2 and the MAPK/p38 signaling pathway in tumor growth and angiogenesis.

**Results:**

BMP2 was highly expressed in HCC. Over-expression of BMP2 was found to accelerate cell proliferation, migration, invasion, microvascular density, and angiogenesis and decrease cell apoptosis in vitro and in vivo. BMP2 silencing exhibited inhibitory effects on HCC cell invasion and angiogenesis. The co-culture system illustrated that HepG2 cells secreted BMP2 in ECV304, and silenced BMP2 in HepG2 cells resulted in the inactivation of the MAPK/p38 signaling pathway, thus suppressing cancer progression, tumor growth, and angiogenesis in HCC.

**Conclusion:**

Taken together, the key findings of this study propose that silencing of BMP2 inhibits angiogenesis and tumor growth in HCC, highlighting BMP2 silencing as a potential strategy for the treatment of HCC.

## Background

Hepatocellular carcinoma (HCC) is a lethal disease that has a high incidence in developed countries [1] and is the third leading cause of deaths in adults across the world [2]. The molecular pathogenesis of HCC is highly complex and heterogeneous in nature, making it particularly cumbersome to find efficient treatment methods [3]. Interestingly, the incidence of HCC has been found to be closely correlated with cirrhosis resulting from chronic hepatitis B virus or hepatitis C virus infection [4]. In addition, owing to the late diagnosis of HCC, patients often exhibit extremely poor survival rates [5]. Recent studies have reported several types of novel treatments for HCC, such as antiviral treatment and immunotherapy [6, 7]. Despite the advancements in surgical techniques and perioperative management, long-term survival rate resulting from surgical resection remains to be especially poor due to the high rate of recurrence and metastasis of HCC [8]. Therefore, it is trivial to elucidate the underlying mechanism and find effective diagnostic and therapeutic approaches for HCC.

A recent study suggested that the bone morphogenetic protein (BMP) family is not solely involved in liver damage response, but also plays a significant role in the promotion of tumor development in HCC [9]. For instance, over-expression of BMP4 was found to be closely related with a poor prognosis of HCC [10]. Another study suggests that BMP2 regulates the promotion of cell angiogenesis, proliferation, and migration via the p38 signaling pathway [11]. In addition, the mitogen-activated protein kinase (MAPK)/p38 signaling pathway is well known to exert a crucial role in balancing cell survival and cell death in various cancers [12]. A previous study further emphasized the important role of the MAPK/p38 signaling pathway on cell apoptosis in acute exacerbation of chronic obstructive pulmonary disease [13]. Moreover, the inhibition of MAPK/p38 signaling pathway is known to serve as a suppressor in cell apoptosis and expression of pro-inflammatory cytokines in human osteoarthritis chondrocytes [14]. Furthermore, the MAPK/p38 signaling pathway can be activated by lysophosphatidic acid, which plays a noteworthy part in the activation of cell adhesion, migration, and invasion in HCC patients [15]. Moreover, a study suggested that activation of BMP2 by hypoxia can promote the activation of the MAPK/p38 signaling pathway in human articular chondrocytes [16]. Based on the aforementioned information, we proposed a hypothesis that BMP2 affects the progression of HCC by regulating the MAPK/p38 signaling pathway and aim to verify this hypothesis to provide some novel insights for HCC treatment.

## Materials and methods

### Ethics statement

Signed informed consents were obtained from all participants, and the experiment was conducted under the approval of the Clinical Trials and Biomedical Ethics Committee of The Second Affiliated Hospital of Nanchang University (2015028). All animal experimental operations were carried out following the convention on international laboratory animal ethics and conform to national regulations.

### Study subjects

A total of 70 patients (39 males and 31 females, aged 28–84 years with a median age of 62 years) diagnosed with HCC after resection at The Second Affiliated Hospital of Nanchang University during September 2015–September 2017 were enrolled in the current study. Subsequently, HCC tissues and adjacent tissues were obtained and stored at − 80 °C for experimentation. According to the Edmondson grading standards, there were 16 cases at stage I, 23 cases at stage II, 21 cases at stage III, and 10 cases at stage IV of HCC patients. In addition, patients were also classified into stage I (*n* = 29), stage II (*n* = 26), and stage III (*n* = 15) according to the tumor node metastasis (TNM) staging published by the Union for International Cancer Control (UICC). Among the included patients, 50 patients presented with intrahepatic tumor metastasis and the remaining did not have intrahepatic tumor metastasis. No included patients underwent radio-chemotherapy or immunotherapy prior to the operation.

HCC cell lines, including MHCC97, Hep3B, HepG2, HCCLM3, and Huh7; human umbilical vein endothelial cell line (ECV304); and normal liver epithelial cell line THLE3 were purchased from the Cell Bank of Chinese Academy of Sciences (Shanghai, China). These cell lines were incubated in Roswell Park Memorial Institute (RPMI) 1640 culture medium (Gibco, Carlsbad, CA, USA) containing 10% fetal bovine serum (FBS) under saturated humidity at 37 °C with 5% CO_2_. Subsequently, the cell lines were subcultured after two rinses with phosphate-buffered saline (PBS), detaching by 0.25% trypsin for 2–5 min and resuspending in 5 mL of Dulbecco’s modified Eagle’s medium (DMEM) (Gibco, Carlsbad, CA, USA) containing 10% FBS.

### Immunohistochemistry

The fresh HCC tissue samples were collected, fixed with 10% formalin, paraffin-embedded, and cut into 3–4 μm slices for immunohistochemical observation. Prior to analysis, the slices were treated with 3% H_2_O_2_ at room temperature for 20 min to dewax and block endogenous peroxidase activity. After 5-min antigen retrieval at 90 °C in an 80% power microwave, the slices were incubated with primary rabbit anti-human BMP2 (dilution ratio of 1:100, ab14933), Caspase-3 (dilution ratio of 1:100, ab2302), and proliferating cell nuclear antigen (PCNA) (dilution ratio of 1:100, ab18197) at 4 °C overnight, followed by incubation with the secondary horseradish peroxidase (HRP)-labeled goat anti-rabbit immunoglobulin G (IgG) (ab6721) at 37 °C for 30 min. All the aforementioned antibodies were purchased from Abcam Inc. (Cambridge, MA, USA). Nucleus staining was then carried out using hematoxylin (C0105, Beyotime Institute of Biotechnology, Shanghai, China) for 30 s, and diaminobenzidine (DAB) (P0202, Beyotime Institute of Biotechnology, Shanghai, China) was employed for color development. Next, the slices were dehydrated using hydrochloric alcohol, sealed with neutral gum, and then observed and photographed under a microscope. The standard for assessing the results of immunohistochemistry was described as follows: the primary antibody was replaced with PBS as the negative control (NC), and known positive slices were taken as the positive control. A total of 5 positive visual fields were selected randomly from each slice (× 400) in order to calculate the ratio of BMP2-positive area to total area.

### Western blot analysis

Once cell confluence reached 80%, a radioimmunoprecipitation assay (RIPA) lysis buffer (BB-3209, Bestbio Science, Beijing, China) was used to extract the total protein from the cells. Total proteins were separated using sodium dodecyl sulfate polyacrylamide gel electrophoresis (SDS-PAGE) and then transferred onto a polyvinylidene fluoride (PVDF) membrane under 80 V. Subsequently, the membrane was incubated with rabbit anti-human BMP2 (ab14933, Abcam Inc., Cambridge, MA, USA) and HRP-labeled rabbit anti-human glyceraldehyde-3-phosphate dehydrogenase (GAPDH, ab9485, Abcam Inc., Cambridge, MA, USA). GAPDH was regarded as the internal reference. After overnight incubation, the membrane was rinsed with phosphate-buffered saline Tween-20 (PBST) for 3 times (10 min/time). Next, the membrane was incubated with HRP-labeled goat anti-rabbit secondary antibody (dilution ratio of 1:10000, Jackson, PA, USA) at room temperature for 1 h. After 3 rinses with PBST (10 min/time), the membrane was placed under an optical luminescence instrument (GE, Ohio, USA) for coloration. After coloration, the Image-Pro Plus 6.0 software (Media, Cybernetics, MD, USA) was employed to analyze the relative protein levels by using gray-scale scanning. The experiment was repeated 3 times in parallel. The other antibodies, including rabbit anti-human BMP2 (ab14933), vascular endothelial growth factor (VEGF, ab69479), VEGF-C (ab135506), matrix metallopeptidase 2 (MMP-2, ab97779), MMP-9 (ab73734), E-cadherin (ab15148), Vimentin (ab137321), extracellular signal-regulated kinases (ERK1/2, ab17942), p-ERK1/2 (ab223500), c-Jun NH2-terminal kinase (JNK, ab208035), p-JNK (ab124956), p38 (ab27986), p-p38 (ab178867), Akt (ab179463), p-Akt (ab192623), and GAPDH (ab9485), were also tested by carrying out the same experimental procedures in cell experiments. Each experiment was repeated 3 times, and all antibodies were purchased from Abcam Inc. (Cambridge, MA, USA).

### Vector construction

Firstly, 3 pairs of BMP2 over-expression sequence (oeBMP2) and short hairpin RNA (shRNA) targeting BMP2 (shBMP2) were designed and synthesized with both Age1 and EcoR I restriction sited attached to both ends, respectively. Subsequently, synthesized oeBMP2 and shBMP2 vectors were detached with both Age1 and EcoR I and then attached to the linear enhanced green fluorescent protein (pGC-FU-GFP) vector which was treated using the same restriction enzymes. The linked products were transferred into the *Escherichia coli* DH5α competent cells (prepared using CaCl_2_ method), and the expression of BMP2 was evaluated using over-expressed or interfered primers via reverse transcription quantitative polymerase chain reaction (RT-qPCR). The positive clones were identified as successfully established oeBMP2 and shBMP2 lentivirus vectors, which were then transfected into 293T cells respectively. Once the green fluorescence from the transfected 293T cells was observed under a fluorescence microscope, the cells were considered to be successfully transfected with the recombinant lentivirus plasmids. Successfully transfected 293T cells were used to produce the virus, which were then extracted and concentrated for further experimentation. The best multiplicity of infection (MOI) value was calculated according to the intensity of green fluorescence under a confocal laser scanning microscope, and the virus titer was measured by fluorescence expression. Finally, the cells were stored at − 80 °C for preservation.

### Cell treatment

HepG2 cells (H) at the logarithmic phase of growth were divided into the following 7 groups: the H_NC group (HepG2 cells infected with lentivirus expressing oeNC), the H_oeBMP2 group (HepG2 cells infected with lentivirus expressing oeBMP2), the H_shNC group (HepG2 cells infected with lentivirus expressing shNC), the H_shBMP2 group (HepG2 cells infected with lentivirus expressing shBMP2), the H_shBMP2 + VEGF group (HepG2 cells infected with lentivirus expressing shBMP2 and injected with commercially available VEGF), the H_oeBMP2 + dimethylsulfoxide (DMSO) group (HepG2 cells infected with lentivirus expressing oeBMP2 and treated with DMSO), and the H_oeBMP2 + SB-239063 group (HepG2 cells infected with lentivirus expressing oeBMP2 and injected with p38 inhibitor, SB-239063). Prior to transfection, the HepG2 cells were inoculated in 6-well plates. Upon reaching 70–80% cell confluence, the cells were infected with lentivirus expressing oeBMP2, shBMP2, oeNC, or shNC in different titers. After 24 h, the infected cells were inoculated with fresh medium containing 500 μg/mL G418 (Gibco, Grand Island, NY, USA), and the culture medium was replaced every 2–3 days based on cell growth conditions. After 12–15 days of transfection, the stably infected and drug-resistant cells were obtained under selection growth with medium containing 500 μg/mL of G418, which was changed every 4–5 days.

### 3-(4,5-Dimethyl-2-thiazolyl)-2,5-diphenyl-2-H_tetrazolium bromide assay

The infected cells at passages 3 to 4 were collected and adjusted to a density of 1 × 10^6^ cells/mL before 2-day incubation in a 96-well plate at a density of 1 × 10^5^ cells/well. In addition to the 7 infected cell samples, additionally, 5 parallel and blank control wells were also set in each group and the incubation was continued. The cells in each well were washed 3 times with DMEM/F-12 culture medium and then mixed with 100 μL of MTT solution (5 mg/mL). After incubation with CO_2_ for 4 h, the MTT solution was discarded. Next, the cells in each well were incubated with 200 μL of DMSO by shaking for 10 min and were allowed to stand for 10 min. The cells were then subjected to a microplate reader to measure the absorbance (*A*) values of each well using an excitation wavelength of 570 nm at 24 h, 48 h, and 72 h.

### Transwell assay

After 48 h of infection, the cells were subjected to Transwell assay using Matrigel (YB356234, Shanghai Yu Bo Biological Technology Co., Ltd., Shanghai, China). Before commencing the treatment, Matrigel was defrosted at 4 °C overnight for equilibrium. The following day, 200 μL of Matrigel gel was diluted with 200 μL of serum-free culture medium at 4 °C, and 50 μL of diluted Matrigel was added to the apical chamber of a plate for Transwell assay and incubated at 4 °C for 2–3 h until solidification. After detachment and counting, the cells were resuspended with complete medium. Afterwards, 200 μL of cell suspension was added to each apical chamber, and 800 μL of culture medium containing 20% FBS was added to each basolateral chamber. Then, the chamber was incubated at 37 °C for 20–24 h. The cells were then rinsed twice with PBS, immersed and washed with formaldehyde for 10 min, washed thrice with tap water, and stained with 0.1% crystal violet. After being allowed to stand for 30 min at room temperature, the cells were rinsed twice again with PBS, after which the cells on the surface were wiped off with cotton. The cells were then observed and photographed under an inverted microscope, and the number of cells was counted at the 0th, 6th, 12th, and 24th hour. The migration experiments were conducted using the same aforementioned methods except that no Matrigel was used to coat the apical chamber.

### Tube formation in vitro

ECV304 cells at passage 3 were inoculated into the basolateral chamber of a 96-well plate at a density of 1 × 10^4^ cells/mL, while the same density of HepG2 cells at passage 3 after transfection was inoculated into the apical chamber. Then, the cells were incubated at 37 °C with 5% CO_2_ in air for 24–48 h, and a polycarbonate membrane (0.4 μm) was employed to separate the apical chamber and the basolateral chamber. The overnight-defrosted Matrigel at 4 °C was distributed into 1.5 mL pre-cooled Eppendorf (EP) tubes (at − 20 °C) according to the requirements. Next, 200 μL of Matrigel was added into each well in a 24-well plate using sterilized pipette tips. The plate coated with Matrigel was then incubated at 37 °C. Meanwhile, a single cell suspension of ECV304 cells that were co-cultured with HepG2 cells was prepared, and the number of cells was counted. After the Matrigel solidified, 1 × 10^6^ cells were transferred into each well and then incubated at 37 °C. The angiogenesis was observed and recorded under a microscope after 4–6 h of incubation.

### Enzyme-linked immunosorbent assay

In order to extract the protein, 50 mg of tissues was placed in a 2.0 centrifugation tube and rinsed with 0.05 mmol/L pre-cooled PBS before being ground with 0.5 mL pre-cooled PBS in a high-speed homogenizer for 2 min. The ground tissues were then centrifuged at 1610×*g* at 4 °C for 10 min to collect the supernatant, and the VEGF concentration was calculated based on the instructions of the ELISA kit (69-99854, Moshake bio, Wuhan, Hubei, China). The absorbance (*A*) value of each well was measured using an excitation wavelength of 450 nm within 3 min employing a microplate reader (Synergy 2, BioTek Instruments, Winooski, VT, USA). With the standard concentration as the horizontal coordinate and the *A* value as the ordinate, the regression equation of the standard curve was calculated. The *A* value was substituted into the equation, and the target protein concentration in the sample was calculated.

### Xenograft tumor in nude mice

Stably infected HepG2 cells (2 × 10^6^) at the logarithmic phase of growth were collected and dispersed into a single cell suspension in PBS after detachment with 0.25% trypsin. The suspension was injected into the subcutaneous part of the right axilla of mice. Depending on the injected HepG2 cells, the nude mice were divided into the H_NC group, H_oeBMP2 group, H_shNC group, H_shBMP2 group, H_oeBMP2 + DMSO group, and H_oeBMP2 + SB-239063 group with 6 mice in each group. The mice were euthanized on the 30th day after inoculation and when the tumor diameter was approximately 2 cm. The fibrous capsule, blood vessel, and the tumor body were removed under aseptic conditions, and the tissues were sliced into 1 mm^3^ cubes after being rinsed with PBS. In addition, 24 female mice (aged 4–6 weeks, weighing 14–16 g) were purchased from the Laboratory Animal Center, Nanchang University (Nanchang, Jiangxi, China). These mice were intraperitoneally anesthetized with 0.6% pentobarbital sodium sulfate. An incision of about 1–2 cm was made under the left ribbed edge, and the abdominal wall was cut in a stratified manner. A tunnel was gently poked under the hepatic capsule with eye tweezers, and normal saline gauze was pressed for a moment to stop the bleeding. The prepared tumor tissues were inserted into the liver of the mouse followed by suture using the “8” shape method. After the tumor was fixed, the liver was placed back in the abdominal cavity, which was sutured intermittently. The maximum diameter (*L*) and the minimum diameter (*W*) of tumors were measured using Vernier calipers on the 7th day after injection. The size of the tumor was measured every 7 days, and the volume of the tumor was calculated using the following formula: *V* = *W*^2^ × *L* × 0.52 [17]. The nude mice were euthanized on the 35th day, and the tumors were extracted, followed by tumor weight measurement. The maximal surface of the tumor tissues of the nude mice was excised without necrotic tissues. The excess part was soaked in 4% neutral formaldehyde solution for fixing overnight. After being paraffin-embedded, the tissues were cut into 10 slices (5 μm) at an interval of 50 μm for further experimentation.

### Hematoxylin-eosin staining

Following tumor isolation from nude mice, the paraffin-embedded tissue slices were dewaxed twice with xylene (15 min/time) and then immersed in anhydrous ethanol twice (5 min/time), 90% ethanol for 5 min, and 80% ethanol for 5 min. Subsequently, the slices were rinsed thrice with PBS (5 min/time), stained with hematoxylin for 3 min, and washed with tap water until turning blue. Next, the slices were differentiated with 1% hydrochloric ethanol for 1 s and washed with tap water until tuning blue. Afterwards, the slices were stained with eosin solution for 1 min, dehydrated with gradient alcohol (70%, 80%, 90%, 100%, 100%, 2 min each time), and cleared twice with xylene (15 min each time) before being sealed with neutral gum. The pathological changes were observed under a microscope (G600, Ze Sheng Yuan Technology Co., Ltd., Shenzhen, Guangdong, China), and images were acquired randomly (× 400) and analyzed using the Morphological Image Analysis System (JD-801, Baoneng Technology Co., Ltd., Xiamen, Fujian, China). The experiment was independently repeated 3 times.

### Terminal deoxynucleotidyl transferase-mediated dUTP-biotin nick end labeling

The aforementioned slices (see the “Xenograft tumor in nude mice” section) were dewaxed and cut into 5 slices. Next, each slice was incubated with 50 μL of 1% protease K diluent at 37 °C for 30 min. Protease-treated slices were first incubated with 0.3% methanol-hydrogen peroxide solution at 37 °C for 30 min to remove the peroxidase (POD) activity and then with the TUNEL solution in a wet box at 37 °C for 1 h avoiding exposure to light, followed by incubation with 50 μL of Converter-POD in a wet box at 37 °C for 30, and incubated finally with 2% DAB for 15 min at room temperature. Once the brown nuclei were apparent under microscope observation, distilled water was added to the slices to terminate the reaction, after which PBS-cleaned slices were subsequently counterstained with hematoxylin, and the reaction was terminated with distilled water. The slices were continuously rinsed three times with PBS (5 min/time) between different reagents. Finally, the slices were dehydrated with gradient ethanol (50%, 70%, 90%, 100%), cleared with xylene, and sealed with neutral gum. Subsequently, the slices were observed under a microscope (× 400), and 5 visual fields in each slice were selected randomly to count the number of positive cells and negative cells. The brown nucleus indicated the apoptotic cells, while blue nucleus coloration indicated normal cells. The ratio between brown cells and blue cells represented the apoptotic index (AI).

### Microvascular density detection

The streptavidin-peroxidase (SP) method was employed for immunohistochemistry in the current study. In brief, the tumor tissues were initially fixed with 10% neutral formaldehyde, dehydrated using gradient ethanol, embedded in paraffin, and cut into 4-μm-thick slices. Next, the slices were dewaxed using xylene and gradient ethanol, rinsed twice with PBS (5 min/time) and twice with distilled water (5 min/time), and then repaired using methanol-hydrogen peroxide for 20 min. Finally, the slices were blocked with 5% normal goat serum and incubated at 37 °C for 45 min before staining. The primary antibody against microvascular density (MVD) (dilution ratio of 1:200) was added to the slices, and then staining was performed according to the instructions of the staining kit. Next, DAB was used for color development. The slices were consequently counterstained with hematoxylin, hydrated, cleared, and sealed with neutral balsam. The primary antibody was replaced with PBS as NC, and the known positive slices were taken as the positive control. While observing the microvessels, the number of microvessels was calculated, and the average value was considered as the MVD value.

### Angiogenesis detection

Fluorescein isothiocyanate (FITC) was used to label Dextra for angiogenesis detection. The location and the increase of microvascular permeability were revealed and quantified by FITC. After a 30-min injection of Evans blue dye (EB), 10% FITC-Dextra (100 mg/kg) was introduced into the tumor-bearing mice via intravenous injection. At the 4th hour after injection, the tumor-bearing mice were euthanized, and the tumor tissues were collected to prepare frozen slices for later observation. At the end, 6–8 visual fields were observed under a confocal microscope to obtain the length and diameter of vessels per unit area in order to calculate the mean values.

### Statistical analysis

The SPSS 21.0 software (IBM Corp. Armonk, NY, USA) was employed for data analyses, and the measurement data were expressed as mean ± standard deviation. Data comparisons between two groups were conducted by *t* test, and comparisons among multiple groups were performed using one-way analysis of variance (ANOVA). A *p* value *<* 0.05 was considered to be statistically significant.

## Results

### BMP2 is positively correlated with angiogenesis in HCC

To investigate the relationship between BMP2 and angiogenesis in HCC, we assessed the expression patterns of BMP2, the correlation of BMP2 with MVD, and the positive expression rate of BMP2 in HCC. As shown in Fig. 1a, a positive correlation was discovered between the positive expression rate of BMP2 and MVD. HCC tissues presented with significantly higher positive expression rate of BMP2 compared to the adjacent tissues (Fig. 1b). Subsequent Western blot analysis results (Fig. 1c) displayed that in comparison with the THLE3 cell lines, the protein levels of BMP2 were significantly increased in the MHCC97, Hep3BLIP-I, HepG2, HCCLM3, and Huh7 cell lines, among which the HepG2 cell line exhibited the highest BMP2 protein expression, and thus HepG2 was selected for subsequent experimentation.

**Fig. 1:** High expression of BMP2 is found in HCC and positively correlates with angiogenesis in HCC. **a** Relative correlation between BMP2 and MVD in HCC. **b** Positive expression rate of BMP2 protein in HCC and adjacent normal tissues detected by immunohistochemistry (× 200). **c** Western blot analysis of BMP2 protein in THLE3, MHCC97, Hep3BLIP-I, HepG2, HCCLM3, and Huh7 cell lines. Data were expressed as mean ± standard deviation, and data between two groups were compared using Student’s *t* test. *p < 0.05. MVD, microvessel density; HCC, hepatocellular carcinoma; BMP2, bone morphogenetic proteins 2

### Silencing of BMP2 restrains cell proliferation, invasion, and migration in HCC

MTT assay and Transwell assay were subsequently conducted in order to measure the cell proliferation, invasion, and migration abilities after infection with lentivirus expressing oeBMP2 and shBMP2 in an attempt to investigate the role of BMP2 that regulates HCC cellular behaviors. These results in Fig. 2a, b showed that the cells infected with lentivirus expressing oeBMP2 presented with significantly enhanced cell proliferation, invasion, and migration abilities, while the cells infected with lentivirus expressing shBMP2 showed a significant reduction in cell proliferation, invasion, and migration. These results suggested that silencing of BMP2 reduced the proliferation, invasion, and migration abilities of HCC cells.

**Fig. 2:** Silencing of BMP2 represses cell proliferation, invasion, and migration in HCC. **a** Cell proliferation ability (measured in OD at 570 nm) in response to over-expression of BMP2 or silencing BMP2 measured by MTT assay. **b** Cell invasion and migration in response to over-expression of BMP2 or silencing BMP2 measured by Transwell assay (× 400). **c** Western blot analysis of MMP-2, MMP-9, Vimentin, and E-cadherin proteins in response to over-expression of BMP2 or silencing BMP2. Data were expressed as mean ± standard deviation, and data between two groups were compared by Student’s *t* test. *p < 0.05. BMP2, bone morphogenetic proteins 2; HCC, hepatocellular carcinoma; OD, optical density; NC, negative control; MTT, 3-(4,5-dimethyl-2-thiazolyl)-2,5-diphenyl-2-H_tetrazolium bromide

In addition, the results obtained from Western blot analysis in Fig. 2c confirmed that the expression of invasion-related genes including MMP-2, MMP-9, and Vimentin was increased upon infection with lentivirus expressing oeBMP2, while that of E-cadherin was decreased. On the contrary, infection with lentivirus expressing shBMP2 resulted in remarkably decreased expression of MMP-2, MMP-9, and Vimentin yet increased E-cadherin expression. These results indicated that BMP2 regulates the expression of invasion-related genes and knockdown of BMP2 reduced HCC invasion.

### Over-expression of BMP2 impedes tumor growth and angiogenesis in HCC

In order to examine whether BMP2 can affect tumorigenicity of HCC cells, we established HCC mouse models. The results of xenograft tumor in nude mice showed that in the H_oeBMP2 group, the tumor was larger and heavier, and the number of HCC cells increased but the apoptotic cells decreased compared with the H_NC group (Fig. 3a, b). In contrast, the tumor was smaller and lighter, while the HCC cells decreased in the H_shBMP2 group when compared with the H_shNC group (Fig. 3a, b). In addition, in the H_shBMP2 group, normal cells were spotted in some region of the tissue, and the number of heterotypic or pyknotic cells was decreased and cell heteromorphy turned to moderate differentiation (Fig. 3c). Furthermore, observation under a laser confocal microscope (Fig. 3d) revealed that the number of vessels was increased markedly when BMP2 was over-expressed, while it exhibited a reduction when BMP2 was diminished. In addition, the results of ELISA (Fig. 3e) illustrated that the protein levels of VEGF were increased remarkably when BMP2 was over-expressed and were reduced when BMP2 was inhibited. Moreover, immunohistochemistry analysis (Fig. 3f, h) showed that BMP2 over-expression resulted in increased positive rates of MVD-CD31 and PCNA and decreased the positive rate of Caspase-3, while the H_shBMP2 group exhibited the opposite changes. The results of TUNEL staining (Fig. 3g) revealed that cell apoptosis was reduced when BMP2 was over-expressed, while enhanced results were apparent when the expression of BMP2 was downregulated. Western blot analysis data (Fig. 3i) suggested that the protein levels of VEGF, VEGF-C, MMP-2, MMP-9, and Vimentin were increased while that of E-cadherin was decreased when BMP2 was over-expressed, and opposite trends in these factors were observed when BMP2 was inhibited. Based on these results, we concluded that silencing of BMP2 repressed the tumor growth, the BMP2 positive rate, and the MVD, thereby inhibiting the angiogenesis in HCC.

**Fig. 3:** Silencing of BMP2 suppresses tumor angiogenesis. **a** Tumor volume and weight after over-expression or silencing of BMP2. **b** Representative image of xenograft tumors. **c** HE staining analysis of pathological changes in response to over-expression or silencing of BMP2 (× 400). **d** Vessel formation in response to over-expression or silencing of BMP2 observed under a laser confocal microscope (× 400). **e** VEGF protein level in serum of nude mice injected with cells infected with lentivirus expressing oeBMP2 or shBMP2 measured by ELISA. **f** Immunohistochemical staining for CD31 (× 400) showing MVD value in response to over-expression or silencing of BMP2. **g** Cell apoptosis in response to over-expression or silencing of BMP2 detected by TUNEL (× 400). **h** Positive rate of Caspase-3 and PCNA in response to over-expression or silencing of BMP2 detected by immunohistochemistry (× 400). **i** Western blot analysis of VEGF, VEGF-C, MMP-2, MMP-9, Vimentin, and E-cadherin proteins in response to over-expression or silencing of BMP2. *n* = 6. Data were expressed as mean ± standard deviation. *p* values were obtained by the Mann-Whitney *U* test. *p < 0.05. HCC, hepatocellular carcinoma; OD, optical density; BMP2, bone morphogenetic proteins 2; HE, hematoxylin-eosin; NC, negative control; VEGF, vascular endothelial growth factor; PCNA, proliferating cell nuclear antigen; MVD, microvessel density; ELISA, enzyme-linked immunosorbent assay; TUNEL, terminal deoxynucleotidyl transferase-mediated dUTP-biotin nick end labeling

### Inhibition of BMP2 secreted from HepG2 inhibits cell proliferation, migration, and vessel formation in vivo by reducing VEGF secretion in endothelial cells

The co-culture of lentivirus-infected HepG2 and ECV304 was conducted to evaluate whether BMP2 affected the angiogenic ability of endothelial cells in HCC. The results (Fig. 4a, c, d) revealed that the cell proliferation, migration, and angiogenic abilities were enhanced upon infection with lentivirus expressing oeBMP2, while all these abilities were restrained upon infection with lentivirus expressing shBMP2. In addition, ELISA was used to detect the protein levels of VEGF, and the results (Fig. 4b) demonstrated that the protein levels of VEGF were increased by BMP2 over-expression and decreased by suppressing BMP2. Moreover, Western blot analysis (Fig. 4e) confirmed that infection of lentivirus expressing oeBMP2 led to increased angiogenesis and elevated protein expression of VEGF, VEGF-C, MMP-2, MMP-9, and Vimentin but inhibited E-cadherin protein expression. On the contrary, reductions in angiogenesis and diminished protein expression of VEGF, VEGF-C, MMP-2, MMP-9, and Vimentin but increased E-cadherin protein expression were observed after infection of lentivirus expressing shBMP2. Notably, the addition of VEGF in co-culture system was found to restore the angiogenesis and tumor formation which were inhibited by infection of lentivirus expressing shBMP2. Altogether, silencing of BMP2 from HepG2 cells suppressed the proliferation, migration, and angiogenic abilities of endothelial cells by downregulating VEGF secretion.

**Fig. 4:** The cell proliferation, migration, and angiogenic abilities of endothelial cells of HCC are suppressed after silencing of HepG2-secreted BMP2. To evaluate the modulatory role of BMP2 in angiogenesis, the HepG2 cells infected with lentivirus expressing oeBMP2 or shBMP2 were co-cultured with ECV304 cells, and VEGF was delivered to HepG2 cells to explore how it functions in a co-culture system. **a** Proliferation of ECV304 cells assessed by MTT assay. **b** VEGF expression patterns in the supernatant of medium evaluated by ELISA. **c** Migration of ECV304 cells tested by Transwell assay (× 400). **d** Angiogenic ability assessed by tube formation assay (× 200). **e** Western blot analysis for expression patterns of angiogenesis-related (VEGF, VEGF-C) and invasion-related (MMP-2, MMP-9, Vimentin, and E-cadherin) proteins. Data were expressed as mean ± standard deviation, and data between two groups were compared by Student’s *t* test. *p < 0.05 compared with the NC group. HCC, hepatocellular carcinoma; BMP2, bone morphogenetic proteins 2; oe, over-expression NC, negative control; VEGF, vascular endothelial growth factor; MTT, 3-(4,5-dimethyl-2-thiazolyl)-2,5-diphenyl-2-H_tetrazolium bromide; ELISA, enzyme-linked immunosorbent assay

### BMP2 activates the MAPK/p38 signaling pathway in endothelial cells of HCC

In order to elucidate the interaction between BMP2 and potential signaling pathways, including the ERK signaling pathway, JNK signaling pathway, MAPK/p38 signaling pathway, and Akt signaling pathway that were related to proliferation, migration, and angiogenesis of ECV304 cells post co-culture with HepG2, we employed Western blot analysis to determine the protein levels of genes related to those signaling pathways in ECV304 cells infected with lentivirus expressing oeBMP2 and shBMP2. The results (Fig. 5a, b) suggested that the protein level ratio of p-p38/p38 was significantly increased when BMP2 was activated but decreased following inhibition of BMP2. No significant changes were observed in the protein level ratios of p-ERK1/2, ERK1/2, p-JNK/JNK, or p-Akt/Akt upon either over-expression or suppression of BMP2. In conclusion, these results demonstrated that BMP2 solely regulated the MAPK/p38 signaling pathway among the 4 aforementioned pathways.

**Fig. 5:** BMP2 regulates the activation of the MARK/p38 signaling pathway in endothelial cells of HCC. **a** Bands of total p38, ERK1/2, JNK, and Akt proteins and phosphorylated proteins in ECV304 cells measured by Western blot analysis after over-expression or silencing of BMP2. **b** Expression of p38, ERK1/2, JNK, and Akt proteins and their phosphorylation extents in ECV304 cells. Relative protein expression values were expressed as mean ± standard deviation, and data between two groups were compared by Student’s *t* test. *p < 0.05. HCC, hepatocellular carcinoma; BMP2, bone morphogenetic proteins 2; NC, negative control; MAPK, mitogen-activated protein kinase

### BMP2 accelerates cell proliferation, migration, and angiogenesis by activating the MAPK/p38 signaling pathway

Based on the results above that BMP2 regulated the MAPK/p38 signaling pathway, we further investigated the mechanism of the MAPK/p38 signaling pathway in HCC in terms of endothelial cell proliferation, migration, and angiogenesis. The results in Fig. 6a–d showed that compared with the BMP2 over-expression alone, inhibition of the MAPK/p38 signaling pathway by SB-239063 resulted in decreased cell proliferation, migration, VEGF protein levels, and angiogenic ability after BMP2 activation. In addition, Western blot analysis results (Fig. 6e) demonstrated that compared with BMP2 over-expression alone, inhibition of the MAPK/p38 signaling pathway led to decreased protein levels of VEGF, VEGF-C, MMP-2, MMP-9, and Vimentin while it increased the protein level of E-cadherin after BMP2 was over-expressed. Thus, we deduced that activation of the MAPK/p38 signaling pathway was involved in the regulatory effects of BMP2 on cell proliferation, migration, and the angiogenic ability of endothelial cells in HCC.

**Fig. 6:** BMP2 enhances cell proliferation, migration, and angiogenic ability via the MARK/p38 signaling pathway. The MARK/p38 signaling pathway was inhibited by SB-239063 when BMP2 was over-expressed to identify the functional significance of MARK/p38 signaling pathway activation in the regulatory effects of BMP2 on ECV304 cell angiogenic ability. **a** Proliferation of ECV304 cells evaluated by MTT assay. **b** VEGF content in the supernatant of medium tested by ELISA. **c** Migration of ECV304 cells measured by Transwell assay (× 400). **d** Angiogenic ability of ECV304 cells by tube formation assay (× 200). **e** Expression of angiogenesis- (VEGF and VEGF-C) and invasion-related (MMP-2, MMP-9, Vimentin, and E-cadherin) proteins measured by Western blot analysis. Data were expressed by mean ± standard deviation, and data between two groups were compared by Student’s *t* test. *p < 0.05. HCC, hepatocellular carcinoma; NC, negative control; MAPK, mitogen-activated protein kinase; VEGF, vascular endothelial growth factor; MTT, 3-(4,5-dimethyl-2-thiazolyl)-2,5-diphenyl-2-H_tetrazolium bromide; ELISA, enzyme-linked immunosorbent assay

### BMP2 promotes angiogenesis in vivo in HCC through MARK/p38 signaling pathway activation

Xenograft tumor in nude mice was conducted to evaluate the functional significance of the MARK/p38 signaling pathway activation in the effects of BMP2 on the tumorigenicity of HCC cells and angiogenesis. The results (Fig. 7a–c) revealed that the H_oeBMP2 + SB-239063 group exhibited smaller and lighter tumor as well as decreased number of HCC cells compared to the H_oeBMP2 + DMSO group. In addition, normal cells were found in some regions of the observed area, while the number of heterotypic or pyknotic cells was decreased, and cell heteromorphy turned to moderate differentiation in the H_oeBMP2 + SB-239063 group. Laser confocal microscopic examination (Fig. 7d) revealed that the formed vessels were decreased in the H_oeBMP2 + SB-239063 group as compared to the H_oeBMP2 + DMSO group. Moreover, ELISA results (Fig. 7e) displayed that the protein level of VEGF was lower in the H_oeBMP2 + SB-239063 group than that in the H_oeBMP2 + DMSO group. Furthermore, immunohistochemistry analysis in Fig. 7f and h showed that compared with the H_oeBMP2 + DMSO group, the positive rates of CD31-MVD and PCNA were decreased while that of Caspase-3 was increased in the H_oeBMP2 + SB-239063 group. TUNEL staining results demonstrated that the AI increased in the H_oeBMP2 + SB-239063 group in comparison with the H_oeBMP2 + DMSO group (Fig. 7g). The subsequent results obtained from Western blot analysis confirmed that the protein levels of VEGF, VEGF-C, MMP-2, MMP-9, and Vimentin were decreased obviously, while that of E-cadherin protein level increased in the H_oeBMP2 + SB-239063 group relative to the H_oeBMP2 + DMSO group (Fig. 7i). Taken together, inactivation of the MAPK/p38 signaling pathway reversed the promoting effects of over-expressed BMP2 on tumor growth, progression, and angiogenesis in HCC.

**Fig. 7:** BMP2 enhances angiogenesis in vivo in HCC through MAPK/p38 signaling pathway activation. The MARK/p38 signaling pathway was inhibited by SB-239063 when BMP2 was over-expressed to identify the functional significance of MARK/p38 signaling pathway activation in the effects of BMP2 on tumor angiogenesis. **a** Tumor volume and weight of nude mice. **b** Representative images of xenograft tumors. **c** HE staining analysis of pathological changes in tumor tissues (× 400). **d** Angiogenesis in tumor tissues under a laser confocal microscope (× 400). **e** VEGF expression patterns in the serum of nude mice detected by ELISA. **f** Immunohistochemical staining for CD31 (× 400) showing MVD value. **g** Cell apoptosis detected by TUNEL (× 400). **h** Positive expression of Caspase-3 and PCNA examined by immunohistochemistry (× 400). **i** Western blot analysis of VEGF, VEGF-C, MMP-2, MMP-9, Vimentin, and E-cadherin protein patterns. *n* = 6. Data were expressed by mean ± standard deviation. *p* values were obtained using the Mann-Whitney *U* test. *p < 0.05; HCC, hepatocellular carcinoma; MAPK, mitogen-activated protein kinase; NC, negative control; VEGF, vascular endothelial growth factor; PCNA, proliferating cell nuclear antigen; ELISA, enzyme-linked immunosorbent assay; HE, hematoxylin-eosin; MVD, microvessel density; TUNEL, terminal deoxynucleotidyl transferase-mediated dUTP-biotin nick end labeling

## Discussion

HCC is a treatment-limited malignancy accompanied by a complex molecular pathogenesis and high mortality [18]. Despite great advancements in treating HCC, these treatments are unobtainable to the majority of the patients, and the physiology of HCC is not well understood, overall limiting the patients’ outcome [19, 20]. Hence, it is of great importance to elucidate the underlying pathological mechanisms related to HCC so as to discover the novel diagnostic biomarkers and therapeutic strategies for HCC. Notably, the BMP family has been previously found to be correlated to the development of HCC [9, 21, 22]. For example, a recent study demonstrated that BMPs such as BMP4 participate in the progression of HCC [23]. We thus explored the role of BMP2 exhibited in regulating the progression of HCC. Eventually, we found that BMP2 was involved in HCC progression through the MAPK/p38 signaling pathway and, furthermore, that HCC cell-secreted BMP2 promotes cell proliferation, migration, invasion, and angiogenesis in endothelial cells by activating the MAPK/p38 signaling pathway.

Initially, we discovered that BMP2 was over-expressed in HCC, and this over-expression promoted the MAPK/p38 signaling pathway-related gene expression. BMP family is derived from the transforming growth factor-beta (TGF-beta) family that possesses binding sites with type I and type II serine-threonine kinase receptors and plays a significant role in transducing signals via Smad and non-Smad signaling pathways [24]. A recent study revealed that upregulation of BMP1 not only contributes to the poor prognosis, but also accelerates the development of gastric cancer, indicating that other BMPs might play a similar role in HCC [25]. In addition, BMP4 was previously revealed to promote cell proliferation by enhancing cell cycle via the ID2/CDKN1B signaling pathway in HCC [26]. Similarly, BMP2 is positively correlated with the stage and development of non-small cell lung cancer [27] and is known to promote cell proliferation and migration via the p38, ERK, and Akt/m-TOR pathways in HCC [11]. MAPK/p38, a significant member of the MAPK superfamily, is induced by varied extracellular stimulation and exerts a significant role in cell apoptosis [28]. Another study suggested that the activation of the MAPK/p38 signaling pathway induced by S100A9 contributes to enhanced cell invasion and growth in HCC patients [29], and additionally, this pathway was realized to also be induced by BMPs, leading to osteoblastic differentiation and mineralization [30]. Moreover, BMP signaling is involved in the p38 signaling pathway in human articular chondrocytes [16]. Thus, these findings and results reflect that BMP2 participates in HCC development via the MAPK/p38 signaling pathway.

The current study also revealed that the protein levels of MMP-2, MMP-9, and Vimentin were increased, while the E-cadherin protein level was decreased as a result of BMP2 over-expression or activation of the MAPK/p38 signaling pathway. The MMP family represents the dominating factors in promoting central nervous system tumor growth, including invasion and spreading, and thereby is of valuable therapeutic importance [31]. In addition, it has been reported that MMP-2 activation induced by the ERK/MAPK signaling pathway contributes to the enhancement of cell proliferation and invasion in endometrial cancer [32]. Moreover, the activation of MMP-9 produced by microRNA-10 was also revealed to lead to increased cell invasion and migration in HCC [33]. Another study further demonstrated that over-expression of MMP-2 and MMP-9 induced by IL-7A can enhance cell migration and invasion via the p38-NF-κB signaling pathway in nasopharyngeal carcinoma [34]. Vimentin, another factor of importance in the current study, as a type III intermediate filament, can be promoted during the epithelial-mesenchymal transition and tumor progression [35]. It has also been found that the upregulation of Vimentin and the downregulation of E-cadherin result in the enhancement of cell migration and tumor metastasis in head and neck squamous cell carcinoma [36]. Interestingly, the expression of MMP-9 is enhanced through the MAPK/p38 signaling pathway in human aortic smooth muscle cells [37]. Additionally, the MMP-2 expression can be increased via the MAPK/p38 signaling pathway in human breast epithelium cell as well [38]. Moreover, a study showed that BMP2 is activated after epithelial injury and results in epithelial dysfunction by downregulating the E-cadherin expression after the occurrence of lung injury [39]. Based on these results, we hypothesized that BMP2 inhibition may suppress cell invasion and migration by mediating the MAPK/p38 signaling pathway and further confirmed the hypothesis via means of Transwell assay. Consistent with our results, a previous study illustrated that the activation of the MAPK/p38 signaling pathway promotes cell invasion and migration in breast cancer [40]. Similarly, another study also highlighted that knockdown of BMP2 serves as a suppressor in cell migration and invasion in gastric cancer by inactivating the PI3K/Akt signaling pathway [41].

Furthermore, the current study uncovered that VEGF protein levels and MVD were increased as a result of BMP2 over-expression or activation of the MAPK/p38 signaling pathway. VEGF is a growth factor that plays significant roles in vascular development and vessel function [42]. Increased VEGF expression and MVD are known to contribute to the angiogenesis of hematological malignancies [43]. Moreover, a recent study confirmed that tissue-type plasminogen activator promotes the expression of VEGF, thereby promoting angiogenesis in endothelial cells by mediating the ERK2/p38 signaling pathway [44]. In addition, BMP over-expression has been suggested to stimulate angiogenesis in bone regeneration by increasing Id1 [45]. Moreover, inhibition of the MAPK signaling pathway has also been suggested to attenuate angiogenesis in zebrafish embryos [46]. Taken together, we demonstrated that BMP2 silencing attenuates angiogenesis by inhibiting the MAPK/p38 signaling pathway.

## Conclusion

In summary, the current study evidenced that BMP2-mediated activation of the MAPK/p38 signaling pathway can promote cell migration, invasion, and angiogenesis, thus accelerating the progression of HCC (Fig. 8). However, further research is warranted in order to accurately identify the effects of BMP2 on the treatment of patients with HCC, in order to advance into an applicable targeted therapy for HCC.

**Fig. 8:** A mechanism map depicting the molecular mechanism of BMP2 in HCC. BMP2 expresses highly in HCC, and the BMP2 secretion from HepG2 into ECV304 cells, then activates the MAPK/p38 signaling pathway, which acts to increase VEGF expression, consequently promoting angiogenesis and tumor growth in HCC

## Data Availability

The datasets generated and/or analyzed during the current study are available from the corresponding author on reasonable request.

## Abbreviations

AI: Apoptotic index
ANOVA: Analysis of variance
BMP: Bone morphogenetic protein
DAB: Diaminobenzidine
DMEM: Dulbecco’s modified Eagle’s medium
DMSO: Dimethylsulfoxide
EB: Evans blue dye
ELISA: Enzyme-linked immunosorbent assay
EP: Eppendorf
FBS: Fetal bovine serum
FITC: Fluorescein isothiocyanate
HCC: Hepatocellular carcinoma
HE: Hematoxylin-eosin
HRP: Horseradish peroxidase
IgG: Immunoglobulin G
JNK: Jun NH2-terminal kinase
MOI: Multiplicity of infection
MVD: Microvascular density
NC: Negative control
PBS: Phosphate-buffered saline
PBST: Phosphate-buffered saline Tween-20
POD: Peroxidase
PVDF: Polyvinylidene fluoride
RIPA: Radioimmunoprecipitation assay
RPMI: Roswell Park Memorial Institute
SDS: Sodium dodecyl sulphate
shRNA: Short hairpin RNA
SP: Streptavidin-peroxidase
TGF-beta: Transforming growth factor-beta
TNM: Tumor node metastasis
UICC: Union for International Cancer Control
